The article "The knowledge map of gender equality in cross-cultural communication: A bibliometric approach" was retracted in 2025. Reason: concerns about the citations.

# The knowledge map of gender equality in cross-cultural communication: A bibliometric approach

**DOI:** 10.1016/j.heliyon.2023.e16324

**Published:** 2023-05-27

**Authors:** Chen Luo, Songyu Jiang

**Affiliations:** a Pass College, Chongqing Technology and Business University, Chongqing, 401520, China; b Rattanakosin International College of Creative Entrepreneurship, Rajamangala University of Technology, Rattanakosin, Nakhon Pathom, 73170, Thailand

**Keywords:** SDG5, Globalization, Interculturalism, Gender issues, Method of bibliometric

## Abstract

It is urgent to solve the gender issues in global cross-cultural communication. Countries worldwide should responsible for achieving gender equality (SDG5). Hence, the study aims to portray the knowledge map of the gender issue in intercultural communication to explore the research status and future potential. The study used *CiteSpace* to conduct a bibliometric method within 2728 English articles on cross-cultural communication and gender equality topics from the *Web of Science (WoS)*. After cluster analysis and time series analysis, this study emphasis the continued attention and increasing trend of publications and elaborates on the critical authors, institutions, and countries of research on this issue. The results introduced Putnick as the dominant author contributed to the topic. The University of Oxford ranked the top1 in the institution cooperation relationship. Europe countries and the United States have made major contributions and influenced Asian and African countries, such as Burkina Faso, North Macedonia, and Kosovo. Gender issues in Asia and Africa are getting much attention. The keyword clusters formed by the authors' cooperation include gender equality, life satisfaction, network analysis, and alcohol use. In addition, childbirth technology, patient safety competition, life satisfaction, capital safety, and sex difference are the key word clustering results of institutional cooperation. At the level of national cooperation, internet addition, risk sexual behavior, covid-19 pandemic and suicidal idea have become the main keywords The results of keyword cluster analysis show that gender role attribute, psychological properties, dating policy, professional fulfillment, and entrepreneurial intention have become the main topics in the current research. The research frontier analysis reflects the importance of gender, women and health. The research on self-efficacy, diversity, image, life satisfaction and choice has become the trend of cross-cultural communication and gender issues. Furthermore, abundant achievement emerged in the subjects of Psychology, Education, Sociology, and Business economics. Geography, Language and Literature, Medicine, and Health industries also have been highly influential in recent years. Therefore, the conclusion suggests the studies of gender issues can be further deepened into more authors, areas, subject and other multiple cooperation sectors.

## 1 Introduction

Cross-cultural communication, as the core concept of the 21st century, has made significant contributions to the development of the world economy, politics, and society [1]. At the same time, it is also an inevitable channel for building a community with a shared future for humankind. The interaction of different races, regions, and countries will lead to the integration of cultures [2]. Cross-cultural communication is extensive content，which is different human groups out of their cultural circles to contact other activities, and this process will produce different cognitions, values, and schemas [3]. Through these cultural exchanges and development, human beings overcome differences and contradictions, achieve cultural integration, and reflect the value of cross-cultural communication [4].

As one of the main aspects of the SDGs, gender issues are not only a local problem in a particular region [5] but also advocate more attention to vulnerable groups such as women, children, and sexual minorities around the world (Schnyder, 2020). Many industries try to solve the troubles caused by gender issues in business, education, politics, and other aspects [6]. Gender equality, sexism, and other topics in different cultural contacts still perform differently in this globalization time [7].

Presently, gender health [8], life satisfaction [9], education [10], internet addiction [11,12], alcohol addiction [13,14], gender roles [15], and psychological problems are crucial gender issues. In cross-cultural communication, dealing with these problems in different cultural backgrounds is our main challenge.

Women's health problems are reflected in many backward areas, pregnancy and diseases caused by sexual life, are not rare [8]. In addition, from the perspective of families, improving the life satisfaction of these women is crucial to their development [9]. The issue of equality in education is no longer new, and women with less education seem more vulnerable to social repression, Internet entry, or alcohol addiction [10]. Therefore, in cross-cultural communication, how to improve gender issues, enhance women's social status, and care about their lives is crucial.

As the leader in cross-cultural research, Europe, the United States, and other developed countries pay attention to the gender issues in their regions [16] and contribute many achievements to gender research in Asia, Africa, and Latin America [17]. In recent years, with the close connection and cooperation between politics, economy, and culture, more and more developing countries have also paid attention to gender issues in intercultural communication, especially in Africa and Latin America [18].

There are four criteria for women's economic activity, political activity, education level, health, and survival. The top five countries that do better gender equality work are Iceland, Finland, Norway, New Zealand, and Sweden. For the past 13 years, Iceland has consistently come to first place with an average score above 0.9, proving that the country does an excellent job of gender equality [18].

Moreover, it may take another 132 years to achieve gender equality worldwide. In the past few years, gender equality actions in various countries have stopped due to the cessation of the COVID-19 pandemic [19]. Especially when schools and childcare institutions are closed due to the covid-19, more women are unemployed and return home to work, or even directly return to the family to support the elderly and take care of children, the pandemic's impact on women is much higher than that of men [20]. Therefore, addressing gender issues in cross-cultural context is urgent. However, some studies discuss gender discrimination [21], gender language [22], and gender equality-related topics in intercultural communication [23].

Gender equality as the SDG5 have received much attention in education and business activities [24]. Gender equality is one of the crucial areas in which the international community measures the degree of sustainable development of the country [25].

In cross-cultural communication, gender studies are gradually declining and becoming marginalized in population studies. The cross-cultural problems caused by gender equality have not disappeared. The challenges faced by SGD5 have not been completely solved. With the new era and new population situation, new problems have emerged. The study of gender issues in cross-cultural communication is of great significance to solving the problems of women and children and promoting the sustainable development of education, the economy, and society [26].

Promoting gender equality in any situation is an urgent moral and social issue and a critical economic challenge [27]. The global economy will also be affected if women, who account for half of the world's working-age population, do not fully realize their economic potential [27]. Gender inequality in cross-cultural communication also indirectly affects investment and population growth [28]. Economic and educational problems caused by gender inequality are particularly prominent in East Asia, sub-Saharan Africa, South Asia, and the Middle East [29].

Table 1 reflects the importance of women's employment and education in cross-cultural communication, a research hotspot. Although the results of bibliometric research on combining the two are not rich, there are not many bibliometric analyses on gender issues and the realization of cross-cultural communication. Table 2 introduces the relevant results of bibliometric analysis.

**Table 1:** The contribution of studying the gender issue in intercultural communication.

	Contribution
Aririguzoh et al. (2022)	Women in different contexts have different discourse rights in cross-cultural communication [30].
Aririguzoh et al. (2022); Alon, T. et al. (2022)	Women's employment in cross-cultural communication will encounter more bottlenecks [31].
Hatayama et al. (2020)	In the digital era, women have more opportunities for employment and can obtain more valuable information through intercultural communication [32].
Shulla, K. et al. (2021)	Equal education will promote a large number of employment, which is an important aspect of current international exchanges [33].

**Table 2:** Introduction to the results of bibliometric analysis of gender issues and intercultural communication.

Topic	Contributions
Gender issues	Gender issues in family business research [34].
	Corporate board gender diversity [35].
	Gender perspectives in tourism studies [36].
	Gender, disability, and Social Identities in tourism Research in Africa [37].
	Trust Gender Biased in E-Commerce [38].
Cross-cultural communication	Forty years of cross-cultural advertising research in the International Journal of Advertising [39].
	Cross Cultural and Strategic Management [40].
	Three decades of the Journal of Teaching in International Business [41].

Table 2 emphasis that the bibliometric analysis of gender issues is carried out in the context of a family business, tourism, company development, and e-commerce. Such analysis is relatively rare in the context of cross-cultural communication research. In addition, the bibliometric analysis of cross-cultural communication also further proves the importance of studying gender issues. There are still many deficiencies in the bibliometric analysis of cross-cultural communication, which only deals with the literature analysis of journals or other topics. Therefore, the research uses bibliometric tools to discuss gender issues in intercultural communication, which is conducive to finding relevant content and research frontiers, thus providing suggestions for future research and other researchers.

Gender inequality in cross-cultural communication hampers progress in reducing unintended pregnancies, high fertility, and child mortality, thereby undermining the well-being of a country [29]. In societies where women are encouraged to take political leadership positions, cross-cultural communication is more gender-balanced [42]. Increasing empirical evidence suggests that cross-cultural communication with high levels of gender inequality carries a greater risk of conflict [28].

Therefore, the study conducted a bibliometric visual analysis of the literature in Web of Science that also contained cross-cultural and gender themes, forming a knowledge graph of the topic. The purpose of the study is to describe the research statue on gender issues in cross-culture in the past five years (2018–2022), moreover, to understand what are the roles of gender equality and intercultural communication to better achieve the SDG5.

Firstly, this article introduces why should visually analyze gender equality in cross-cultural communication and explains its significance for sustainable development. After that, the paper discussed the impact of cross-cultural communication and gender equality on sustainable development through literature analysis. Next, the methods of data acquisition and visual analysis are described. The fourth part explains the publication trends, author cooperation, institutional cooperation, national cooperation, keyword co-occurrence, and research trends. Moreover, this part portrayed the related knowledge map. Finally, the paper summarizes the full text and puts forward the contribution and value of the research.

This is almost a new attempt to analyze gender equality and cross-cultural communication based on visual analysis to explore its significance for sustainable development. The research aims to understand the current situation and future of gender research in cross-culture, as well as to find the current hot spots and trends in cross-cultural gender research to attract more scholars to pay attention to this topic. It also provides relevant advice on addressing gender issues in intercultural communication.

## 2 Literature review

### 2.1 Cross-cultural communication and sustainable development

Cross-cultural communication in the age of globalization and digitalization is almost an entirely new concept that affects the communicative activities of human society [43]. Meanwhile, it also can be problematic because the underlying conceptual elements and words used to describe its features may be largely culture-dependent [44]. The present study was conducted to understand similarities and dissimilarities in the concept of Cross-culture communication in different regions. However, in the process of achieving the goal of sustainable development, intercultural communication plays an important role [42].

Intercultural communication in education is a new challenge in the context of education for sustainable development [45]. Cultivating the intercultural communication ability of higher education students is a factor in achieving the goal of sustainable development [46]. Therefore, at the level of education internationalization, the complexity of language determines the degree of cross-cultural communication [47]. The promotion of intercultural communication has become an essential factor in achieving the sustainable development of education [48]. In addition, improving the intercultural communication ability of teaching staff has also positively impacted education for sustainable development [45].

The promotion of sustainable development by intercultural communication is not only reflected in the field of education but also has a significant impact on the sustainable development of tourism [49]. Thailand has begun to pay attention to how language perception and intercultural communication can promote the sustainable development of tourism [50]. The perceived demand of local communities for English is a factor that attracts tourists from Europe and the United States [51]. Therefore, in encouraging the sustainable development of tourism, Cross-cultural training is also of considerable significance, which involves preparation time and actual communication time [52].

Similarly, in fashion design, cross-cultural communication enables countries and nations to learn from each other about design concepts, processes, and styles, forming a positive interaction of the sustainable development of the industry's culture [53]. By cultivating the global capabilities of designers, it is helpful to enhance the diversification and continuous cooperation in the field of global design [53]. At the same time, cross-cultural communication plays an essential role in guiding the communication between the village and the urban system and, thus, in the sustainable development of rural areas [54].

Therefore, it has become a trend for intercultural communication to promote sustainable development [25]. Although there are more fields and researchers to join in this section, it is necessary to understand the research clues of intercultural communication affecting sustainable development to provide new ideas and contribute to sustainable development in the era of globalization.

### 2.2 Gender equality and sustainable development

Gender equality is essential in pursuing the SDGs, which emphasize the equal rights of women, children, and sexual minorities in social development and promote harmony between people and society [55]. Gender issues remain acute in many countries in the 21st century [21]. However, evidence points to cross-national convergence and persistent (or even growing) heterogeneity in women's status when different aspects of gender inequality [56]. To make sense of this contradiction, Cole et al. (2018) examine how culture moderates the relationship between economic development and gender inequality [56].

Gender equality itself is part of the concept of sustainable development. Shannon, Jansen [8]provided evidence for why gender equality in science, medicine, and global health matters for health and health-related outcomes. Alarcón et al. (2019) explored the interconnections between the Sustainable Development Goals (SDGs) and tourism from a gender perspective [57]. Scarborough et al. (2019) show that gender attitudes have more than one underlying dimension and that these dimensions have changed at different rates over time [58]. In light of the sustainability goals introduced through the UN's 2030 Agenda for Sustainable Development, Levin et al. (2019) present a model to systematically address gender mainstreaming in transport planning [59]. Lau et al. (2021) provide an overview of four common gender assumptions and offer four suggestions for a more scholarly pursuit of gender equality in climate change policy and practice [60]. These achievements fully demonstrate the importance of gender equality for sustainable development. Moreover, the evidence on the relationship between gender equality and sustainable development in the Middle East and North Africa shows that adolescents have a substantial demographic dividend advantage and are likely to make more contributions to economic growth and development [61]. The goal of sustainable development is characterized by gender intersection. Girls are an essential part of demography on the way to achieving SDGs, especially the mainstreaming of gender equality into all SDGs [62]. Regarding anthropological tendency, gender equality also has particular legal value [63]. In addition, the study on gender equality from Nigeria also confirmed that gender equality is conducive to achieving the expected sustainable development of the country [64].

In summary, many studies in the past five years have focused on cross-cultural communication and gender equality. Moreover, many results have focused on the relationship between the two and sustainable development. However, the discussion of gender issues in intercultural communication is still not deep enough, and the fields involved are not extensive enough. Some research trends are already in analyzing cross-cultural communication research [2]. However, almost no results have paid attention to gender research in intercultural communication. In particular, these findings rarely focus on the inspiration of gender equality in intercultural communication for sustainable development. This paper tries to analyze gender research in cultural communication based on many academic achievements, analyze research trends, authors, institutions, national cooperation, discipline distribution, and keyword contributions, provide corresponding suggestions for the development of this field, and promote sustainable development.

## 3 Research method

Web of Science (WoS), as one of the primary databases of bibliographic research, covers cutting-edge research in many disciplines and is a high-quality tool commonly used in bibliometric analysis [65]]. The study used the advanced search function in WOS, based on the research results after 2018, and carried out the output of the following three search formats.

The first search formula (1) requires that the literature subject contain both cross-cultural and gender English articles, revealing 1236 results.

The second search format (2) requires that the literature subject include cross culture and gender Articles in English, totaling 1258 results.

The third search query (3) requires the literature subject to include *cross-culture, cross-cultural, or cross cultural, and gender* within English articles.

A total of 2728 results delete the articles bookmarked in the previous search. The result obtained in the final search formula 3 is 1324. As one of the main tools for visual analysis of knowledge graphs, CiteSpace has made an essential share for analyzing research status and trends in various fields [66]. The study imported these results (3818) into CiteSpace, divided them, as shown in Table 3, left only the article-like results, and finally analyzed the 2728 results for knowledge graph analysis. That includes discussions of the timing, author, institution, and keywords to reveal the current status and future of gender research in intercultural communication. Based on these articles, the study of different categories of clustering and time series analysis in the “title + topic + abstract” by software. Dig out different clusters under author, institution, country, and subject categories, and introduce the development and relationships of related topics through time series.

(1) (((TS=(cross-cultural)) AND TS=(gender)) AND DT=(Article)) AND LA=(English)
(2) (((TS= (cross culture)) AND TS=(gender)) AND DT=(Article)) AND LA=(English)
(3) (((((TS=(cross-cultural)) OR TS= (cross culture)) OR TS= (cross cultural)) AND TS= (gender)) AND LA=(English)) AND DT=(Article) (TS = topics; DT = literature type; LA = language)

**Table 3:** Cite Space deduplication results analysis.

Total Records Found: 3818
3818 Article
–
Total Unique Records (Article): 2728
Duplicates: 181
Discarded: 1090

The research first uses three retrieval formulas to obtain the data in WOS and then uses Citespace to perform de-duplication processing. Then, it uses 2728 articles as the primary reference data for the next step of the analysis. In the next part, the research analyzes the year of publication, author cooperation, institutional cooperation, national cooperation, discipline cooperation, and keyword co-occurrence of the research on gender equality in cross-cultural communication by bibliometric method. Almost every part determines the clustering relationship in the knowledge map through cluster analysis to find the current status and future research clues of cross-cultural communication and gender equality.

## 4 Data analysis

### 4.1 Years of publications

Cite Space conducted an annual analysis of 2728 results and found that since 2018, Table 4 suggests the number of posts published has gradually increased each year, from 2018 (438) to 2021 (675). The study of gender in cross-culture has developed better and better in the academic community in recent years, and many results have promoted the development of this research. Because 2022 has only passed half a year, the number of literatures have reached 368, and the study is expected to be 2022. By the end of the year, the number of related posts may exceed 700. Therefore, the study of gender issues in cross-culture is in line with the current research hotpots and trends. The outcome reflects the importance of gender issues in cross-culture in human social development, and observing gender issues from a new cultural communication perspective is more conducive to solving gender-related social problems in the world and promoting the realization of SGD5 (gender equality).

**Table 4:** Trends of cross-cultural and gender research publications.

Year	No. publication
2018	438
2019	593
2020	654
2021	675
2022	368

### 4.2 Knowledge maps of author cooperation

The analysis of authors' cooperative knowledge map aims at mining authors who have made outstanding contributions to the research in the field and interpreting the cooperation between authors through relationship nodes [67].

By the cooperative author cluster computing, 5 clusters appeared. Moreover, the study concluded the related authors of six clusters of collaborative knowledge atlas. Putnick made a related effort around the theme of the argument method. WHO and Taber have contributed significantly to gender equality. Brooks emerged under the life satisfaction cluster, and the network analysis part of Chang et al. was relatively active in the middle. Alignment methods and gender equality became the most central topics of discussion.

As the most significant author collaborative theme clustering, the *alignment method* appeared on average in the 2015, with a size of 36. Gender equality appeared on average in the 2018, which was 21 in size, becoming the second cluster. Similarly, as a topic of discussion in 2019. *life satisfaction* was 19. *Network analysis* appeared on average in 2018. *Alcohol use* appeared on average in 2016. Table 5 explicitly introduces the keywords formed by different clusters and their sizes. Therefore, the topics and hot-pots of academic concern are different in different periods. The scholars who explored this topic in 2018–2019 were the most numerous and concentrated.

**Table 5:** Cluster size and keywords by author cooperation.

Cluster ID	Size	Year	Keywords	Cluster Keywords
0	36	2015	body appreciation; collective action intention; country-level gender equality; unit-weighted score	alignment method
1	21	2018	gender equality; authenticity scale; double standard; sex difference; accepting external influence	gender equality
2	19	2019	life satisfaction; university student; other variable; self-care activities; psychological well-being	life satisfaction
3	15	2018	network analysis; age group; present study; fcv-19s item; factor structure	network analysis
6	10	2016	alcohol use; college alcohol belief; low-risk drinking; high level; occupational class	alcohol use

The authors from European and American countries seem to be more interested in the issue of intercultural communication and gender equality [68]. They have pushed this topic into the research field worldwide. Intercultural communication and gender equality are indeed an idea that involves the well-being of all humanity [69]. Hence, Table 6 illustrated top-10 authors based on the CiteSpace contribution index.

**Table 6:** The main authors contribute to the topic of cross-culture and gender.

Count	year	Source
16	2016	Putnick (2016)
13	2014	WHO (2014).
11	2020	Brooks (2020)
11	2018	Taber (2018)
10	2015	Brown (2015)
10	2014	Hair et al. (2014)
9	2018	Falk (2018)
7	2017	Ryan (2017)
7	2016	Rodriguez (2016)
7	2014	Davidov et al. (2014)

Putnick (2016) contributed significantly to the study of gender in intercultural communication, highlighting it 16 times in the knowledge graph. Secondly, the Global Status Report on *Violence Prevention* released by the WHO (2014) became the second largest source of contribution, highlighted 13 times in the knowledge graph. By analogy, Brooks (2020) and Taber (2018) highlighted 11 times, Brown (2015) and Hair et al. (2014) highlighted ten times, Falk (2018) highlighted nine times in the knowledge graph, Ryan (2017), Rodriguez (2016) and Davidov et al. (2014) appeared seven times each in the knowledge graph. Hence, the authors became among the top ten contributors to gender studies in intercultural communication and continue to advance research beyond 2018.

### 4.3 Knowledge maps of institutional cooperation

The atlas of institutional cooperation can reflect the leading institutions that study gender equality in cross-cultural communication worldwide. Through the visual analysis of institutional cooperation, the theme and development of cooperation between institutions can emerge [67].

Fig. 1 describes the ten highest-cited universities, the first of which is the University of Oxford, cause the strength of this institution equals to 3.3, followed by the University of Amsterdam, with strength of 2.63, Univ Kansas (2.3), the University of Manchester (2.3), and the University of Melbourne (2.19). However, their research was mainly in 2018–2020, followed by Charles univ Prague (1.97), Shiraz univ med SC I (2.74), Univ Southampton (2.24), Brown University (1.74), and Stockholm univ (1.74) continue to contribute to research.

**Fig. 1:** Top 10 institutions with the strongest citations burst.

The study used the “title + keyword + abstract” under the CiteSpace agency cooperation map for cluster analysis. A total of 10 clusters were generated: childbirth technology, patient safety competence, life satisfaction, marital satisfaction, sex difference, alcohol use severity, emerging adult, network analysis, psychogenic nonepileptic seizure, and middle eastern countries.

The University of Washington and the University of Southern Denmark are still working on children and patients. Zhejiang University's attention to marine life is also continuing around 2022. Loyola University has also contributed to the study of gender roles. In terms of annual distribution, since 2018, the University of Washington, the University of British Columbia, the University of Auckland, the University of Hong Kong, and the University of Amsterdam have been working on these types of research. The University of Chicago, Harvard University, and the University of Edinburgh have also gradually emerged research results in 2019. Even more surprising is that relevant research in Asian and African countries will promote gender research across cultures, such as Korea University, Sudan University, Wuhan University, and Nigeria University, around 2020. From the overall point of view, the contribution of universities in Europe and the United States to this topic is relatively high. In recent years, universities in Asia and Africa have also been influenced by cross-cultural and gender studies in European and American universities, making essential contributions to adults, the Middle East, and pathology.

### 4.4 Knowledge maps of country cooperation

The analysis of the national cooperation map aims to make it easier to identify the major countries that have contributed to the thematic research. Through the analysis of the national cooperation knowledge map, it is mainly to decrypt the development held by different countries at a particular time and the research alliances formed with other nations. Moreover, this analysis can also reflect the main themes of different countries [67].

Six clusters were formed using the clustering method of *“keyword + title + abstract”* based on national cooperation. Pakistan and Italy have corresponding results under the clustering of addictive networks around 2018, which will also impact this topic in 2022. Spain, Guinea, Bissau, and Qatar have made efforts since 2018 the study risk of sexual behavior in Aruba. Senegal has received continued influence from previous countries in the last year or two discussions on this topic.

Furthermore, India, Australia, Sri Lanka, Tanzania, and Vietnam contributed more to the dunning-Kruger effect around 2018. Brunei, Rwanda, and other countries continued to make achievements. The research results of the dunning-Kruger effect show that developing countries research is more prominent under this cluster, especially in the Asian and African regions.

European countries such as Finland and Portugal have led the study of the intodermqol questionnaire in the early stages. In the past two years, Uzbekistan, Nigeria, Angola, and other countries have also appeared in the clustering of the intodermqol questionnaire in 2022. Montenegro emerged as a representative in clusters. The covid-19 pandemic is a hot topic that has been studied continuously since 2020. China and Togo are more representatives in this cluster.

As for suicidal ideation, studies focused on it almost until 2020, with few national studies observing suicidal ideation in 2021 and 2022 clustering. At the same time, the study of gender in cross-culture was more the result of developed countries in Europe and the United States in the early stage, and they made more contributions to this, from the perspective of time, the impact on the later research is also beyond doubt. However, after 2019, developing countries dominated by Asia and Africa paid more attention to the problem of sex ratio in their own countries.

Fig. 2 explains that *Burkina Faso, North Macedonia, and Kosovo* are particularly prominent. From 2018 to 2020, Morocco and Suriname with strength of 0.43 have become the region of most significant concern 2020, which means that the world is currently paying particular attention to the gender issues in these countries across cultures. It is not difficult to see that these regions are mainly African, which fully reflects the plight of the African region in this regard and the contribution made by the world to this.

**Fig. 2:** Top 5 countries with the strongest citations burst.

The study used CiteSpace to analyze the Centrality of the National Cooperation Atlas, which we chose centrality ranks in the top ten. Centrality is the number of shortest paths through points in a network and a measure of the size of connections played by nodes in the overall network [70]. Moreover, the counts can reflect the quantity of countries contributing to the topics. Nodes with significant centrality are relatively easy to become critical nodes in the network. Table 7 reveals that the United States with 768 counts and the centrality is 0.2, England (271), China (262), Germany (182), Spain (164), Canada (147), Australia (134), Italy (134), India (133), Pakistan (95), and Iran (95) have become significant forces in studying cross-cultural and gender topics. In other words, developed and super-populated countries (China, India) in Europe and the United States have contributed significantly to this topic and impacted cross-cultural and gender studies worldwide.

**Table 7:** The main countries contribute to the topic of cross-culture and gender.

Count	Centrality	Year	Country
768	0.02	2018	USA
271	0.03	2018	England
262	0	2018	Peoples R China
182	0	2018	Germany
164	0	2018	Spain
147	0.02	2018	Canada
134	0.02	2018	Australia
133	0.01	2018	Italy
101	0.02	2018	India
95	0	2018	Pakistan
95	0.01	2018	Iran
90	0.01	2018	Turkey

### 4.5 Knowledge maps of keywords

Keyword co-occurrence analysis is the foremost step of visual analysis and one of the most powerful data processing functions of Cite Space [67]. The keyword map analysis aims to reveal the main topics and hotspots that may be involved in gender equality in cross-cultural communication. To some extent, the keyword map allows researchers to interpret the current research situation and get clues for future research.

The study uses the clustering method of “keyword + title + abstract” to form 9 clusters at the keyword analysis level. These clusters are expanded gender role attitude, psychometric properties, dating violence, professional fulfillment, entrepreneurial intention, social skill, physical activity, interpersonal deviance, and work-family practices.

There is a vast number of nodes in 2018, indicating that the discussion of this topic in 2018 is particularly prominent, and this year focuses on topics such as self-efficacy, adults, children, age, women, experience, cultural behavior, gender differences, discrimination, etc. The research of 2018 continued to advance in 2019, and the Chinese emerged. In the same year, keywords such as violence, assault, fear, marriage, ethnic culture, adulthood, children, and other words also existed.

After that, the research pushed the topic into new areas, such as life satisfaction, medals, illness, personal characteristics, wisdom, and other keywords gradually appeared. Keywords include variance structure analysis, structural equation models, capital, and workforce. Inspire our research on this topic to enter the management field in 2022, primarily using quantitative research methods to solve related problems.

Keyword strongest citation burst emphasizes the development track of relevant topics and can provide reasons for future research because keyword emergence suggests the most popular research direction in the field [67].

Fig. 3 continued to analyze highlighting high-citation keywords and selected the top 25 high-citation keywords. The study found that in 2018–2019, validation factor analysis became the highest citation, meaning that much research on gender in cross-cultures comes from a quantitative perspective and that academia is trying to address the correlated factor problem. Secondly, keywords such as material use, collectivism, individualism, and commitment declare that the study of this topic involves multiple fields, especially in terms of culture. Highly cited keywords include job satisfaction, business, employee, and occupation. Gender studies in cross-cultural contexts have contributed to economic management, especially human resource management. In the past two years (2020–2022), it has been revealed more from the psychological perspective, and we can get some clues from keywords such as life satisfaction, image, self-efficacy, death, and diversity, hence, the academia should continue focus on the psychological study in the context of gender issue in intercultural communication.

**Fig. 3:** Top 25 keywords with the strongest citations burst.

Table 8 introduces the keyword with the most significant number of nodes as gender, which existed 422 times. The study only selected keywords with a node number greater than 100, women, health, gender differences, behavior, attitudes, prevalence, culture, models, and validity. Among them, which means gender issues in cross-culture, women's issues, in particular, are particularly prominent in terms of gender discrimination, health, and psychological aspects such as behavior and attitudes. Among them, perception has the strongest centrality (0.03), indicating that perception has the most significant impact, reflecting that the study of gender issues in cross-cultural concepts is a hot topic. On the other hand, the keywords selected are all from 2018, which means that these studies in 2018 have a great inspiration for subsequent attempts and are also crucial.

**Table 8:** The main keywords to the topic of cross-culture and gender.

Count	Centrality	Year	Keywords
422	0.01	2018	gender
177	0.02	2018	women
176	0.01	2018	health
175	0.01	2018	gender difference
156	0.01	2018	behavior
155	0.01	2018	attitude
142	0.01	2018	prevalence
131	0.01	2018	impact
126	0.01	2018	culture
117	0.03	2018	perception
107	0.01	2018	model
104	0.01	2018	validation

### 4.6 Knowledge maps of research subjects

The strongest citation bursts analysis of subject categories emphasizes the main research disciplines involved in cross-cultural communication and gender equality, which can provide more opportunities for the integration of disciplines for future research and also make up for the lack of research in some disciplines [49]. Fig. 4 analyzes the highest cited discipline, finding that geography, rehabilitation, philosophy, psychology, biology, Chemistry, and primary health care were frequently cited until 2020. After 2020, linguistics, health policy and services, and medical informatics became the leading disciplines of cross-cultural and gender studies.

**Fig. 4:** Top 10 subject categories with the strongest citations burst.

Table 9 extracted disciplines with more than 100 nodes. The counts in Table 9 represents the number of literatures contributed by each discipline. It is clear that psychology (622) and SSCI (588) have absolute advantages and have become the primary disciplinary sources of cross-cultural and gender studies. In addition, the fields of environment, health, business, and medical care have also contributed a lot to this topic. Moreover, the field of education (147) is among the main contributing subjects. From the perspective of Centrality, the node of SSCI (0.91) is the most prominent and clear. However, psychology also has a certain degree of correlation with other disciplines (0.25). However, the Psychology, Multidisciplinary social science citation index (SSCI) is relatively independent and almost challenging to relate to other disciplines.

**Table 9:** The main keywords to the topic of cross-culture and gender.

Count	Centrality	Year	Subjects
622	0.25	2018	Psychology
588	0.91	2018	Social science citation index (ssci)
240	0.15	2018	Public, Environmental & Occupational Health
198	0.15	2018	Business & Economics
177	0	2018	Psychology, Multidisciplinary we social science citation index (SSCI)
163	0.03	2018	General & internal medicine
147	0.16	2018	Education & educational research
138	0.07	2018	Social sciences - other topics
136	0.03	2018	Psychiatry
133	0.01	2018	Public, Environmental & Occupational health we science citation index expanded (SCI-expanded)
112	0.15	2018	Humanities citation index
107	0.01	2018	Science & technology - other topics
100	0.06	2018	Environmental sciences & ecology

## 5 Discussion and conclusion

Cross-cultural has almost become a theme in the current process of building a community with a shared future for humanity [71]. The challenges faced by management [72], behavior [73], psychology [74], social media [75], cross-cultural communication opportunity [31], and its importance to the development of the times have long been important topics in scientific research. As gender issues are an essential aspect of the SDG5, gender issues will inevitably be discussed in intercultural communication [76].

Gender roles in cross-cultural communication [28] (abuse of women and children, female roles, feminism), gender language [77] (women's voice, female expression, children's language), and gender literature have become the main aspects of gender issues worldwide. Nonetheless, few studies have summarized and reviewed these achievements.

This article belongs to the primary stage of bibliometric analysis. Therefore, the study is only a study of gender equality in cross-cultural communication, revealing the critical areas involved in this topic between 2018 and 2022, as well as the relevant research status, providing more ideas for cross-cultural communication and gender equality research, and guiding a specific direction. The results of bibliometric analysis of gender equality in the context of intercultural communication, although gender issues are crucial to sustainable development.

The bibliometric analysis of cross-cultural communication has made some breakthroughs, but the research content is relatively simple, mainly from the perspective of communication science, and hardly combines the gender issues. Therefore, the results have new significance for sustainable development. Therefore, the innovation in research ideas and methods has broken through the previous research's focus on gender issues only. Both qualitative and quantitative research is the basis for this paper to obtain conclusions and inspire future research.

We are conducive to sorting out the development trend of cross-cultural and gender research, hot topics, the current status of the author, institutional cooperation, and the direction of future research.

The achievements of gender issues study in cross-cultural context had increased year by year, indicating that the topic has gradually attracted more and more attention worldwide. From the national cooperation map perspective, the current Asian and African regions in the cross-cultural gender problem is still more severe.

In the early stage, the developed countries and world-class universities have made important achievements on this topic. They continue to affect the attention of developing countries such as Asia, the Middle East, Africa, Latin America, and other developing countries to pay attention to gender issues in the past two years. It will take a long time to achieve gender equality, and gender equality is only one aspect of gender issues. From the perspective of national cooperation, the United States, the United Kingdom, and China have contributed the most to cross-cultural and gender research, focusing on gender issues in their own countries or other regions. These countries have highlighted their interest in SDG5 attention.

Moreover, among these countries, the University of Washington, Harvard University, Zhejiang University, the University of Amsterdam, and the University of Southern Denmark have become the main force of cross-cultural and gender studies and have led higher education institutions in Asia and Africa to devote themselves to this aspect of research. The study illustrates from the thematic atlas that gender issues in current cross-cultural contexts are represented in many categories. Such as gender roles, marriage, violence, alcohol addiction, sexual assault, child abuse, working in family life, life satisfaction, employment, entrepreneurship, social skills, psychological problems, and much more.

The focus of different periods and different scholars are not exact. In the past two years, the research has paid more attention to gender topics from the perspectives of psychology, business and economics, education, linguistics, and medicine, such as women's employment and life satisfaction, work self-efficacy, death, abuse, sexual health, gender language literature and other issues.

These results inspire researchers to enter the field of research from many aspects and further focus on gender issues in intercultural communication in the context of a covid-19 pandemic. Specifically, researchers can discuss cross-cultural gender issues from the fields of education, business, and politics rather than simply discussing the relevant content of their own cultures.

Furthermore, the study encourages more scholars to conduct comparative research on gender issues in different cultures so that more fields can pay attention to gender issues in different cultures. The results will address society's negative development due to gender discrimination or roles.

On the other hand, in discussing gender issues in intercultural communication, while solving the topic of women and children, we should pay more to the issue of sexual minorities in cross-cultural cultures. Furthermore, more and more countries have positively solved the problems of sexual minorities from the aspects of laws, policies, and insurance have individual results to instruct and guide different societies to pay attention to these groups. Nevertheless, from this analysis of the study literature, there is no clue that sexual minorities in cross-cultures are receiving sufficient attention.

Hence, the study implicates the introduction of relevant gender policies in cross-cultural communication, including gender issues in education, gender protection and respect topics in work, and the need for continuous support in the policy. Comparing gender policies in different countries is one of the critical methods to promote gender studies in intercultural communication. Developed countries should pay more attention to women's issues in Africa and the Middle East, especially gender discrimination in cross-cultural communication. At the same time, cooperation institutions in different countries should strengthen the research alliance of cross-cultural communication and gender equality and further realize SDG5 through education, enterprises, and employment.

Bibliometric analysis results lead researchers to recognize the significance of studying intercultural communication and gender equality for SDG5.

However, there are also some defects. Only the data from WoS can be used as the dataset. In the future, relevant content may be mined from more databases, including reliable documents in Scopus, SSCI, and ProQuest. In addition, the research results of the past five years mainly reflect the current research status, so the research and exploration of the context of this topic are from the perspective of diachronic development, especially its origin and development process. If we examine intercultural communication and gender equality from a macro perspective, future research must focus on the whole development process of the topic. Finally, in data generation, the query topic is particularly critical. The research should probably do more synonym retrieval or similar phrase retrieval to expand the search scope, which is also a problem that should be paid attention to in future research.

In the future, the other researchers could contribute more diachronic, comparative, and empirical research to address cross-cultural and gender issues in different fields, continue serving the SDG5, and pursue more opportunities to respect and love people and lives after the Covid-19 pandemic.

This article explains the current hot topics of cross-cultural and gender studies from the perspective of literature atlas analysis and the scholars, institutions, and countries working on the topic. The study introduces the positive trend of the development of this topic year by year and encourages more subject areas to participate in the discussion of this topic, not only psychology, management, pedagogy, language, and literature, but also other disciplines closely related to cross-culture should pay attention to this aspect. Gender issues manifest themselves differently at different times and regions, so there is still a long way to go to solve this problem.

The research has surprisingly discovered that traditional gender inequality is still very prominent in many countries, especially the social status of women in low-income countries, which should attract the attention of all sectors. Gender issues in cross-cultural communication show diversity and seriousness, mainly in alcohol abuse, addiction to the Internet, sexual health, and education inequality. Inequality in employment is more likely to attract attention in recent years. Cross-cultural communication in the digital era of the 21st century provides a new way to solve gender problems. Therefore, it has become crucial to pay attention to the psychological problems and sustainable development issues related to women's technology, life satisfaction, image, and entrepreneurial intention. If our research is to catch up with the unpredictable requirements of the times, we need more diachronic, comparative, and empirical research to address cross-cultural and gender issues in different fields, continue serving the Sustainable Development Goals of gender equality, and pursue more opportunities to respect and love people and lives after the Covid-19 pandemic.

## Data availability statement

The authors do not have permission to share data.

## Institutional review board statement

Not applicable.

## Informed consent statement

Not applicable.

## Declaration of competing interest

The authors declare that they have no known competing financial interests or personal relationships that could have appeared to influence the work reported in this paper.
